# Bearing Strength of Concrete-Filled Steel Tube Reinforced with Internal Transverse Stiffened Bars under Axial Compression

**DOI:** 10.1155/2022/1704544

**Published:** 2022-02-21

**Authors:** Nan Li, Yajun Xi, He Li, Guangxi Zhang, Tao Ren, Xinhao Mu

**Affiliations:** ^1^College of Resources, Shandong University of Science & Technology, Taian 271019, China; ^2^Tai'an Engineering Construction Standard Cost Office, Taian 271000, China

## Abstract

A new type of square concrete-filled steel tubular (SCFST) column is proposed, which is characterized by transverse stiffened bars inside the steel tube to improve the effective constraint performance of the concrete core. The experiment of this kind of composite material under axial compression was carried out. The results showed that the bearing capacity of the SCFST column reinforced by internal transverse stiffened bars increased by 4.5%-15% than that of the ordinary SCFST column. The transverse strain is smaller than the SCFST column. As the diameter of the reinforcement increases and decreases the spacing of bars, the axial load bearing capacity increased. The transverse strain of the member decreased obviously. It is noted that the confinement performance of the concrete core of this type was improved to some extent. At the same time, based on the unified theory, the simplified calculation formula of axial compression bearing capacity is derived.

## 1. Introduction

The outer steel tube of the concrete-filled steel tube structure can effectively improve the restraint internal concrete, and the concrete under the transverse restraint of the steel tube is better in the three-dimensional compression state, so that the concrete can better exert its compressive performance [1–5]. As a kind of steel-concrete composite system, the SCFST column has been widely used in the structure because of its convenient connection, high flexural bearing capacity, and beautiful appearance. Based on the above characteristics, square steel tube concrete in civil engineering theoretical research and engineering applications has become more widespread in recent years [6–12]. Kong and Moon [13] studied the carrying capacity and energy dissipation of SCFST columns under long-term axial load. Uy [14] studied the mechanical properties of the short columns under the combined action of axial compression and bending moment. Susantha et al. [15] proposed an approximate formula for the axial compression-strain of confined concrete in concrete-filled steel tubular columns with different cross-sections. Liu et al. [16] studied axial compression bearing capacity of rectangular steel tube high-strength concrete short column. The load capacity obtained by the experiment was compared with the calculated values of EC4, AISC, and ACI. Liang et al. [17] proposed a method of nonlinear analysis of fibrous elements to predict the ultimate strength and ductility of thin-walled steel columns made of concrete subject to local buckling. Normal stress redistribution in the steel sheet appears after the local buckling. It is also proposed that the ductility and section performance of reinforced concrete square columns can also be described by two performance indexes. Dundu [18] carried out axial compression tests on 29 square concrete-filled steel tubes, obtained the axial compressive strength, and proposed a two-stage equation to simulate the calculation formula of short columns and medium to slender columns. Dai and Lam [19] studied the structural fire behavior of a series of concrete-filled steel tubular (CFST) short columns with four typical column cross-sections under standard fire conditions. The experimental results show that the circular section of CFST columns has the best structural fire behavior. Based on this, the design simplified formula of the concrete column under high temperature is put forward. Evirgen et al. [20] conducted axial compression tests on 48 concrete-filled steel tubular columns with different variables and studied and analyzed the influences of width-thickness ratio, compressive strength of concrete, and column geometric parameters on axial bearing capacity, ductility, and buckling performance of concrete columns. Ellobody and Young [21] proposed a way for calculating the bearing capacity of square stainless steel reinforced concrete tubular columns. Raed et al. [22] proposed a method for calculating the axial load capacity of concrete-filled steel tubes through the experimental results of the axial compression performance of square stainless steel pipes. Many experts and scholars have put forward various measures and structures to enhance the restraint effect of square steel tubes on core concrete in the SCFST structure. Alfarabi et al. [23] studied the axial carrying capacity of the stainless steel short column without or filled with concrete. It is improved by welding carbon steel reinforcement on the inner surface of the circular hollow stainless steel pipe and the stainless steel pipe concrete short column. The change of adding stiffeners in square section concrete-filled steel tubular members is studied by Fang [24], and the eccentric compression test of members is carried out. It is found that the stability and ultimate strength of columns are improved. The reinforced concrete column with external restraint reinforcement ring and internal reinforcement is studied by Alrebeh [25]. The experiment shows that compared with the member with external reinforcement ring or internal reinforcement, the combined use is more effective to improve the structural performance of short column members. To further improve the performance, the spacing of internal reinforcement can be reduced and the number of internal reinforcement can be increased. Li et al. [26] proposed a new composite member with I-shaped carbon fiber reinforced polymer wrapped inside to strengthen square steel tube short columns and carried out a bidirectional bending test on it. The results show that the new short column has good bearing capacity and ductility in the biaxial bending test. Alatshan et al. [27] reviewed the existing literature on stiffened concrete-filled steel tubular and proposed a method to systematically review the relevant knowledge of stiffened concrete-filled steel tubular in the existing literature. Zhu et al. [28] proposed the connection method of the outer diaphragm using perfobond ribs (PBL) to strengthen concrete-filled square steel tubes (CFSST). The test shows that this innovative connection method improves the load transfer and deformation of the joint.

From the above studies, it is not difficult to find that the outer steel tube is less constrained to the internal concrete core of the SCFST column. Therefore, in order to better promote restraint of foreign steel tubes to concrete, more effective restraint measures should be developed and researched.

In this paper, a new type of SCFST column is presented. The main structural feature of the column is that some transverse reinforcing bars are welded on the inner wall of the square steel tube to strengthen the restraint of the core concrete of the square steel tube; at the same time, the local stability of square steel tube walls is strengthened, and the ultimate bearing capacity and deformation capacity of the SCFST column under axial pressure are effectively enhanced. Axial load capacity and ductility are analyzed; from the perspective of unified theory, a formula for a theoretical evaluation of load bearing capacity of SCFST with internal transverse stiffened bars is proposed.

## 2. Experimental Programme

### 2.1. Specimen Fabrication

A total of 10 specimens were tested under compression, including one square concrete steel tubular stub column and nine SCFST with internal transverse stiffened bars. Before the experiment, in order to facilitate the observation of the deformation of the specimen, a square was drawn with chalk on the test block in advance. All specimens were made of 6 mm thick steel plates with a height of 600 mm and a side length of 200 mm. The stiffener diameters are 4 mm, 6 mm, and 8 mm, respectively, and the stiffener length is 180 mm. Internal transverse reinforcement spacing is 50 mm, 75 mm, and 100 mm, respectively. The steel plate material is Q235B, and the transverse bar is HPB335. The typical section is shown in Figure 1, and all specimens are given in Table 1.

### 2.2. Material Properties

All the samples were made of a 6 mm thick steel plate. A part of steel was cut directly from the steel plate of the square steel pipe, and the standard tensile test strip of steel was made for the material property test. Tables 2 and 3 describe the mechanical properties of steel and reinforcement, respectively. Meanwhile, concrete-filled square steel tube specimens were poured; 3 pieces of concrete cube specimens with side length of 150 mm were made for the material performance test. The average compressive strength of concrete cube specimens with curing age of 28 days is 31.6 MPa.

### 2.3. Experiment Setup

This test uses the YAW-3000A electrohydraulic Servo pressure testing machine as shown in the figure. The load is carried out by the way of hierarchical axial loading [29]. Place the sample in the center of the tester. A steel block is fixed at the upper and lower ends of the specimen to prevent local failure near the load surface. At the same time, ensure that the centroids of the base, sample, and steel block are on the same vertical line. The experimental loading equipment used in the study is shown in Figure 2.

The main measurement content includes the longitudinal and transverse strain of the specimen, the axial pressure of the specimen, and the value of axial compression deformation. The longitudinal strain of the column is attached to the 4 outer surfaces of the steel pipe column, 3 on each surface, and the positions are located at 1/4, 1/2, and 3/4 of the height of the specimen. The transverse strain is measured by the horizontally attached strain gauges. Paste 3 on the 4 outer surfaces of the steel pipe column. The positions are located at the middle height of the test piece and distributed at 1/4, 1/2, and 3/4 of the cross-sectional width. The outer surface of the test piece is longitudinal and transverse. The position of the strain gauge is shown in Figure 3.

In the elastic phase, the value of the control load at each step is about 10% of the value of the limit load. Each loading step takes 3-5 minutes. When the value of the load increases to 85% of the calculated limit load, the loading speed is reduced until failure. The test loading time for each specimen is about 2 hours.

## 3. Experimental Results

### 3.1. Failure Mode

The failure mode of specimens is shown in Figure 4. Both samples showed local buckling of the steel pipe. For the specimens of B0, local buckling of steel pipes is in the height direction, but for specimens of B1-B9, the local buckling is a little or not obvious. The failure mode of SCFST specimens is mainly the outward bulging and buckling of steel tubes at the top and middle, and the outer bulging area and size are large. The failure of SCFST with internal transverse stiffened bars columns mainly occurs at the top. At the same time, there is a slight bulging and buckling at the middle and upper parts of SCFST, but it is not particularly obvious. The size is 5~10 mm. In the same group of specimens, with the decrease of the spacing of transverse stiffeners, the degree of external bulging tends to decrease, indicating that the increase of transverse reinforcement on the pipe wall can effectively delay the buckling of the steel plate.

### 3.2. Comparison of Load Bearing Capacity

According to the experimental observation and the load-displacement curves of specimens, as shown in Figure 5, these compression specimens usually have three stages from the beginning of loading to the failure of the specimen.

In the first stage, at the beginning of loading, the specimens are in an elastic phase as seen from the load-strain curves. There are no obvious changes in the steel tube.

In the second stage, when the load is up to 85% of the ultimate capacity, the surface deformation of the square steel tube appears in some parts and the specimens show elastic-plastic behavior. At this stage, the local buckling of the steel tube appears at first near the upper end of the specimen, then develops to the middle of the specimen, and the phenomenon of local buckling is gradually obvious. When the load reaches the limit load, the local buckling deformation of the steel pipe wall is obvious.

At the last stage, when the load reaches the ultimate load, the internal concrete is destroyed, the load-carrying capacity of the specimen decreases rapidly, and the displacement increases continuously.

As seen from Figure 5, the load summit of the ordinary SCFST column specimen (B0) is much smaller than that of the other 9 specimens (SCFST with internal transverse stiffened bars column). It is indicated that the transverse stiffened bars can play an active role in SCFST. With the different configurations of transverse stiffened bars, the increase in the axial load bearing capacity is different.

From Figures 5(a)–5(c), it can be seen that when the diameter of the transverse steel bars is constant, reducing the spacing of the transverse steel bars will increase the axial load bearing capacity, but the magnitude of the increase varies. Traditional SCFST specimens have a small peak point displacement; SCFST with internal transverse stiffened bars column has better ductility due to the stiffened steel bars. The peak point displacement is large, and the final displacement can reach 10-15 mm. When the spacing of the transverse stiffening ribs remains unchanged at *S* = 100 mm and the diameter changes, the bearing capacity only increases by 0.8% to 1.8%; when the spacing of transverse stiffeners is *S* = 75 mm, the ultimate bearing capacity is only increased by 1.6%~3.3%; when the spacing of transverse stiffeners is *S* = 50 mm, the change of diameter increases the bearing capacity by 1.7%~4.9%.

According to the above analysis, for the SCFST with internal transverse stiffened bars column, the effect of improving the bearing capacity of SCFST with internal transverse stiffened bars column through the change of reinforcement diameter is not obvious; the change of the spacing of transverse stiffeners is conducive to improve the bearing capacity of SCFST with internal transverse stiffened bars column. Decreasing the spacing of transverse stiffeners is more effective than increasing the diameter of stiffeners. With the larger diameter of bars and the smaller spacing of transverse bars, the increase of axial supporting capacity is more obvious. The axial supporting capacity of all specimens is shown in Table 4.

As seen from Table 4, the load bearing capacity of the SCFST column with transverse stiffened bars is better than that of SCFST columns. In all specimens, the maximum increase amplitude is 15%; the smallest increase reached 4.5%; this is mainly due to the weak confinement of the square steel tube on the core concrete. When transverse stiffened bars are welded on the inside steel tube, it can strengthen the restraint effect of the square steel tube on concrete, make the concrete in the core area get better compression from three directions, and improve the bearing capacity of concrete. It is noted that the transverse stiffened bars inside the steel tube can play an important role in promoting the load bearing capacity of SCFST columns.

### 3.3. The Amount of Steel in Concrete-Filled Steel Tube

The amount of steel of specimens is shown in Table 5.

#### 3.3.1. The Effect of the Variation on the Bar Diameter

According to the data in Table 5, we can know that the steel consumption of the square steel reinforced concrete column is 2.3%, 3%, 4%, 5.1%, 6.6%, 9.5%, 9.1%, 11.7%, and 16.8%, respectively. And the corresponding increase in bearing capacity is 3%, 5%, 7%, 4%, 9%, 12%, 6%, 12%, and 15%, respectively. Remaining the spacing of 100 mm unchanged, when the diameter of the transverse stiffened bars changed from 4 mm, 6 mm, and 8 mm, the corresponding increase in the amount of steel was from 2.3%, 5.1%, and 9.1%, while the corresponding increase in the bearing capacity changed from 4.5%, 5.3%, and 7.1%; remaining the spacing of 75 mm unchanged, when the diameter of the transverse stiffened bars changed from 4 mm, 6 mm, and 8 mm, the corresponding increase in the amount of steel was from 3%, 6.6%, and 11.7%, while the corresponding increase in the bearing capacity changed from 6.7%, 9.9%, and 11.5%; remaining the spacing of 50 mm unchanged, when the diameter of the transverse stiffened bars changed from 4 mm, 6 mm, and 8 mm, the corresponding increase in the amount of steel was from 4%, 9.5%, and 16.8%, while the corresponding increase in the bearing capacity changed from 8.4%, 13.3%, and 15%.

#### 3.3.2. The Effect of the Variation on the Bar Spacing

Remaining 4 mm of the diameter of bars unchanged, when the cross bar spacing is reduced from 100 mm to 75 mm and from 75 mm to 50 mm, the corresponding increase in the amount of steel is 2.3% and 4%, respectively. The increase of the bearing capacity is 4.5% and 8.4%, respectively. Remaining 6 mm of the diameter of bars unchanged, when the cross bar spacing is reduced from 100 mm to 75 mm and from 75 mm to 50 mm, the corresponding increase in the amount of steel is 5.1% and 9.5%, respectively. The increase of the bearing capacity is 5.3% and 13.3%, respectively. Remaining 8 mm of the diameter of bars is unchanged, when the cross bar spacing is reduced from 100 mm to 75 mm and from 75 mm to 50 mm, the corresponding increase in the amount of steel is 9.1% and 16.8%, respectively. The increase of the bearing capacity is 7.1% and 15%, respectively. Under the condition of constant reinforcement diameter, when the transverse reinforcement spacing is reduced from 100 mm to 50 mm, the bearing capacity of the transverse reinforced concrete column is about 4% higher than that of the concrete-filled steel tubular column.

It can be seen from Figure 6 that the influence of the increase of bearing capacity by the decrease in the bar spacing is more obvious than the increase of the bar diameter in the SCFST with the internal transverse stiffened bars column. In Figure 5(b), the changes of load capacity are more obvious when spacing from 75 to 50 mm. Therefore, in the practical application, the ultimate bearing capacity of SCFST columns can be improved by reducing the internal transverse bar spacing firstly when the same amount of steel is used.

### 3.4. Comparative Analysis of Transverse Strain

The transverse strain of three sections on all specimens is shown in Figure 7.

As seen from Figure 7, due to the confinement effect of transverse stiffened bars, transverse strain is smaller than that of the SCFST column; meanwhile, with the decrease of spacing of stiffened bars, transverse strain becomes smaller. The change of transverse strain affected by the diameter of the stiffened bar is not obvious, stiffened bars are confined to the core concrete in the steel tube, and the confinement effect of SCFST with internal transverse stiffened bars column is strengthened. The change trend of transverse strain on each section of the column is basically the same.

### 3.5. Comparison of Concrete Failure Forms inside the Square Steel Tube

In order to observe the failure of the steel pipe wall and the concrete, the outer steel plate was cut off after the test. It was found that the main form of failure of the concrete near the square steel pipe wall in the specimen was crushing (Figure 8). For the specimens without transverse stiffeners, the concrete collapse is serious. The concrete is crushed obviously at the outer drum of the outer steel plate; the cracks have extended to the inside of the core concrete, indicating that the specimens are damaged. But the concrete collapse in the square steel tube with transverse stiffeners is not obvious. Only a small number of concrete fragments are found falling off at the location of the transverse reinforcement. After removing the concrete on the outer surface, the size of the cracked area became smaller, indicating that the steel pipe and the concrete are reliably combined through the transverse steel bars. The restraining effect is obvious, and its bearing capacity has a certain degree of improvement.

## 4. Simplified Calculation Method

In order to facilitate the calculation and be easy to apply in practical engineering, the form of the formula should be simplified as far as possible. In the simplified formula proposed in this paper, the bearing capacity of concrete under the restraint of internal transverse reinforcing steel bar and square steel tube is taken as the basic calculation part, and the confinement factor of the transverse reinforcing steel bar and SCFST has been considered. A large number of studies show that the restraint effect of SCFST on the core area is an important factor to improve the bearing capacity of SCFST, so the confinement effect coefficient *ξ* is introduced. This coefficient is related to the strength of steel, the cross-sectional area of the steel tube, the strength of concrete, the cross-sectional area of core concrete, and so on. The calculation formula of *ξ* is shown in (4). With the unified theory based on the concrete-filled steel tube, Zhong [8] put forward a composite compressive strength design formula:

(1) $$\begin{array}{c} N_{0}=\left(1.212+B\xi +C\xi^{2}\right)f_{ck}A_{sc}, \end{array}$$

where

(2) $$\begin{array}{c} B=0.1759\frac{f_{yk}}{235}+0.974, \end{array}$$

(3) $$\begin{array}{c} C=-0.1038\frac{f_{yk}}{20}+0.0309, \end{array}$$

(4) $$\begin{array}{c} \xi =\frac{A_{S}/A_{C}}{f_{y}/f_{c}}, \end{array}$$

(5) $$\begin{array}{c} A_{SC}=A_{S}+A_{C}. \end{array}$$

In this paper, according to the calculation model of the above formula, the axial bearing capacity of the SCFST column with internal transverse stiffened steel bars is calculated as follows:

(6) $$\begin{array}{c} N_{0}=\left(A_{1}+B_{1}\xi +C_{1}\xi^{2}\right)f_{c}A_{sc}. \end{array}$$

Based on (6), the bearing capacity of the SCFST column with internal transverse stiffened steel bars can be calculated, as shown in Table 6, and the value of the test results and the test values of the bearing capacity of the test are calculated by the method of the two regressions:

(7) $$\begin{array}{c} \frac{N_{0}}{f_{c}A_{SC}}=A_{1}+B_{1}\xi +C_{1}\xi^{2}. \end{array}$$

The regression coefficient, *A*_1_ = 0.25, *B*_1_ = 2.185, *C*_1_ = −0.1987, *R*^2^ = 0.96.

Substituting Formula (7),

(8) $$\begin{array}{c} N_{0}=\left(0.25+2.185\xi -0.1987\xi^{2}\right)f_{c}A_{sc}. \end{array}$$

It should be noted that this paper analyzed the parameters of the range as follows.

Width thickness ratio *B*/*t* = 33.3‐50, yield strength of steel *f*_*y*_ = 235 MPa, and compressive strength of concrete *f*_*c*_ = 14.3 MPa (concrete strength grade C30). By*ξ* = *A*_*s*_*f*_*y*_/(*A*_*c*_*f*_*c*_) ≈ 4*t*′*f*_*y*_/(*bf*_*c*_), the coefficient range is approximate to *ξ* = 1.3 − 2.3.

The bearing capacity of the specimens calculated by Formula (8) and the test piece pressure bearing capacity obtained from the experiment are recorded in Table 6.

From Table 6, the average value of *N*_0_/*N*_1_ is 1.0, the standard deviation of *N*_0_/*N*_1_ is 0.015, and the coefficient of variation of *N*_0_/*N*_1_ is 0.015. The test results are basically consistent with the calculation results, which can be used in engineering practice.

## 5. Conclusion

In this paper, the variation law of axial compression capacity of the SCFST column with internal transverse stiffened steel bars is studied. Through the comparison of test results, the correlation between column bearing capacity and steel quantity is analyzed, and the following conclusions are drawn:

1. By adding transverse reinforcement, the constraint effect of steel tube wall on concrete is improved, and the local buckling of steel tube wall outward is effectively delayed, and the interaction between steel tube and core concrete is strengthened
2. The existence of transverse reinforcement enhances the hoop sleeve effect and increases the bearing capacity of the SCFST column with internal transverse stiffened steel bars by 4.5~15%. At the same time, the strain of each cross-section of the SCFST column with internal transverse stiffened steel bars decreases and distributes more evenly along the height direction
3. When the amount of steel used is the same, the bearing capacity of the new structure column can be improved more effectively by decreasing the spacing of transverse stiffeners than by increasing the diameter of reinforcement
4. When the diameter of the steel bars is the same, the bearing capacity of the SCFST column with internal transverse stiffened steel bars increases significantly with the decrease of the spacing of the transverse steel bars; when the spacing of the transverse steel bars is the same, the bearing capacity of the SCFST column with internal transverse stiffened steel bars slightly increases with the increase of the diameter
5. Based on the unified theory of SCFST, the simplified formula for calculating the pressure bearing capacity of the SCFST column with internal transverse stiffened steel bars is proposed

## Figures and Tables

**Figure 1:** The specimen.

**Figure 2:** Test device.

**Figure 3:** Layout of measuring points.

**Figure 4:** Failure mode of specimens.

**Figure 5:** Comparison of load-displacement curve.

**Figure 6:** The influence between the change of steel and load bearing capacity.

**Figure 7:** Comparison of transverse strain of columns.

**Figure 8:** Damage of concrete in square steel tubes B0 and B4.

**Table 1:** The dimension of specimens.

Specimen	Width (mm)	Height (mm)	*t* (mm)	Diameter (mm)	Length (mm)	Spacing (mm)
B0	200∗200	600	6	None	None	None
B1	200∗200	600	6	4	180	100
B2	200∗200	600	6	4	180	75
B3	200∗200	600	6	4	180	50
B4	200∗200	600	6	6	180	100
B5	200∗200	600	6	6	180	75
B6	200∗200	600	6	6	180	50
B7	200∗200	600	6	8	180	100
B8	200∗200	600	6	8	180	75
B9	200∗200	600	6	8	180	50

**Table 2:** Mechanical properties of steel.

Plate thickness (mm)	Yield strength (MPa)	Tensile strength (MPa)
6	228	310

**Table 3:** Mechanical properties of steel bar.

Diameter of steel bar (mm)	Yield strength (MPa)	Tensile strength (MPa)
4	353	460
6	345	430
8	332	420

**Table 4:** Bearing capacity of specimens.

Specimens	Bearing capacity (kN)	Increasing amplitude (%)
B0	2112	—
B1	2177	4.5
B2	2230	6.7
B3	2270	8.4
B4	2197	5.3
B5	2310	9.9
B6	2400	13.3
B7	2240	7.1
B8	2350	11.5
B9	2440	15

**Table 5:** Comparison of steel consumption.

Specimen number	Weight of steel tube (kg)	Weight of steel bars (kg)	Total amount of steel (kg)	Steel ratio
B0	21.9	0	21.9	1
B1	21.9	0.50	22.4	1.023
B2	21.9	0.64	22.54	1.033
B3	21.9	0.92	22.82	1.043
B4	21.9	1.12	23.02	1.051
B5	21.9	1.44	23.98	1.066
B6	21.9	2.08	23.89	1.081
B7	21.9	1.99	23.89	1.095
B8	21.9	2.56	24.46	1.117
B9	21.9	3.69	25.59	1.168

**Table 6:** Comparison of bearing capacity between theory and test.

Specimen	*ξ*	Value of test *N*_1_ (kN)	Value of calculation *N*_0_ (kN)	*N*_0_/*N*_1_
B1	2.020	2177	2204	1.01
B2	2.040	2230	2220	1.00
B3	2.061	2270	2236	0.99
B4	2.071	2197	2244	1.02
B5	2.127	2310	2287	0.99
B6	2.170	2400	2320	0.97
B7	2.150	2240	2305	1.03
B8	2.245	2350	2376	1.01
B9	2.317	2440	2429	1.00

## Data Availability

The data supporting the results of this study are available in the article.
